This article has been retracted.

# Safety Risk Assessment of Tourism Management System Based on PSO-BP Neural Network

**DOI:** 10.1155/2021/1980037

**Published:** 2021-09-20

**Authors:** Wenru Guo

**Affiliations:** ^1^School of Tourism and Urban-Rural Planning, Zhejiang Gongshang University, Hangzhou, Zhejiang 310018, China; ^2^School of Tourism Management, Xinyang Agriculture and Forestry University, Xinyang, Henan 464000, China

## Abstract

With the development of science and technology, system management is gradually applied to tourism management. How to correctly assess the security risks of the tourism management system has become an important means to maintain passenger information. The security risk index of the travel management system is input into the PSO-BP network as a sample, and the corresponding risk value of the index is used as the network output. The results show that the error results, accuracy (96.53%), training time (216 s), number of iterations (275 times), and convergence speed are all better than traditional BP network. The relative error of PSO-BP network (0.32%) is better than that of BP network, with 300 iterations, and the error is close to 10–5. The average evaluation accuracy of *S* based on PSO-BP network is 99.72%, and the average time consumed is 2.512 s. It is superior to the evaluation model based on fuzzy set and entropy weight theory and the evaluation model based on gray correlation analysis and radial basis function neural network. In conclusion, the security risk assessment of the tourism management system based on PSO-BP network can effectively assess the security risk of the tourism management system.

## 1. Introduction

With economic and technological developments and the continuous improvement of people's living standards, tourism has become a common leisure way for people to relieve pressure and enjoy their minds and bodies, and the tourism industry has brought about rapid development [1]. With the proliferation of tourism-related data and information, the traditional tourism management model has gradually replaced Internet technology, and the tourism management system has shifted to management [2]. While networks provide convenience to users, they also increase the security risks of travel management systems. Effective and scientific assessment of system security risks is an important way to ensure network information security [3]. A BP neural network (BPNN) is a multilayer forward network based on error backpropagation, consisting primarily of an input layer, several hidden layers, and an output layer. It has strong nonlinear fitting capabilities and has some practicality in classifying, identifying, and calculating risk values [4, 5]. BPNN can classify any complex pattern and has excellent multidimensional function mapping capabilities. This greatly improves network classification and network recognition capabilities and has powerful application effects in solving nonlinear problems [6]. However, in the BPNN network's self-learning process, changes in thresholds or weights make BPNN training more prone to the situation of local minimal solutions and reduce the accuracy of risk values in tourism management systems [7, 8]. At the same time, the BPNN network requires more training time, the corresponding slow convergence speed, and poor real-time control performance [9]. Particle swarm optimization (PSO) is used to improve BPNN to improve BPNN calculation accuracy. This speeds up BPNN training and reduces the chances of the latter going to the limit.

Ramesh et al. [10] verified the effectiveness of the back propagation neural network model in prediction of stock returns. Parwez et al. [11] trained a neural network prediction model with anomalous and nonanomalous data to highlight the influence of anomalies in data while constructing the intelligent model; this can greatly improve the accuracy of neural networks. Wang et al. [12] have used evolutionary algorithms to improve traditional BP neural network algorithms to prevent particles from falling into locally optimal solutions. Researchers such as Ai and Yang [13] have proposed a machine learning method based on a support vector machine optimized by a particle swarm optimization algorithm and applied it to cost prediction of environmental governance. Wen and Yuan [14] have introduced random forest algorithms and particle swarm optimization algorithms into the construction of commercial sector carbon dioxide emission prediction models to establish new network prediction models based on BP neural networks. The results show that the model can accurately predict carbon dioxide emissions in the commercial sector. Jiang et al. proposed [15] the particle swarm optimization algorithm in combination with the BP neural network algorithm to establish predictive models and predict the cost of product remanufacturing based on data-driven methods. The results show that the model has high prediction accuracy. Hao and Zhu [16] established a Levenberg Marquardt Backpropagation (LMBP) neural network and used it to predict the quality of polyamide 66 gears.

Particle swarm optimization algorithms such as be used for training neural networks and for co-designing PSO training neural network software and hardware [17]. Zhang et al. [18] obtained a global optimal parameter-optimized data-driven framework through the PSO algorithm and proposed a data-driven detection technology for laser welding defects based on real-time spectrometer signals. Dehghanbanadaki et al. [19] estimated the unconstrained compressive strength of natural fillers using two feed-forward artificial neural network models trained by particle swarm optimization algorithms and BP neural network algorithms. In the process of investigating safety risk assessments and early warning mechanisms in building engineering, researchers such as Ma et al. [20] have managed cloud security based on the scalable theory of distributed computing to quantitatively assess the safety status of construction sites. When studying the mechanism of security sharing strategies in information sharing systems, scholars such as Ss et al. [21] proposed a new corporate information sharing framework from the perspective of information system security and implemented the optimal level of information sharing strategies. Researchers such as Zhang et al. [22] have conducted 28 activities to conduct social ecosystem risk assessments and ecosystem service stress assessments at the mouths of subtropical coasts of Brazil to directly generate supplies and cultural ecosystem services for habitat risk assessments. Scholars such as Terzi used Bayesian networks, agent-based models, and system dynamic models to assess multiple risks in mountainous areas [23–25].

In summary, there have been many studies in recent years on artificial neural networks, BP neural networks, particle swarm optimization, and system security risk assessment, but there is a lack of relevant research on security risk assessment of tourism management systems. The BP neural network algorithm is optimized through the particle swarm. Therefore, this article proposes a security risk assessment technology for tourism management systems based on the PSO-BP neural network to help people quickly assess the security risks of tourism management systems.

## 2. Safety Risk Assessment of Tourism Management System Based on PSO-BP Neural Network

### 2.1. System Security Risk Assessment Based on PSO-BP Neural Network

BPNN has adaptive learning functions [26]. The feedback propagation mechanism constantly adjusts the weights of the network parameters, reducing the difference between the output vector and the expected vector.

First, the least squares method is used to plan the formula for the 3-layer BP neural network, and then the number of hidden layer neurons is determined by continuously adjusting the experimental parameters (Figure 1).

(1) $$\begin{array}{c} h={\left(0.43mn+0.12m^{2}+2.54n+0.77m+0.35\right)}^{1/2}+\alpha . \end{array}$$

Formula (1) is the formula for calculating the number of neurons *h* in the hidden layer. The number of neurons in the input layer and the output layer is *n* and *m*, respectively; *α* is a constant, and *α* ∈ (0,9). At the same time, BPNN uses limited accounting to calculate the error between the predicted result and the actual expected value.

(2) $$\begin{array}{c} E=\frac{1}{2}\sum_{j=1}^{J}{\left(d_{j}-Y_{j}\right)}^{2}. \end{array}$$

Formula (2) is the error calculation formula of BPNN network, where the mean square error is *E*; the expected output value and the actual output value of the output layer *j* are expressed as *d*_*j*_ and *Y*_*j*_ in turn; *J* refers to the number of neurons in the output layer. BPNN network completes the input and output of the network mainly through neurons.

(3) $$\begin{array}{c} y_{j}=f\left(\sum \omega_{ji}x_{i}+\theta_{i}\right). \end{array}$$

In formula (3), *y*_*j*_ and *x*_*i*_ refer to network output prediction results and network input sample data, respectively; the connection weight is *ω*_*ji*_; the threshold value is *θ*_*i*_, which reflected the connection strength between neurons; and the transfer function is *f*.

(4) $$\begin{array}{c} f\left(x\right)=\frac{1}{1+e^{-x}}. \end{array}$$

Equation (4) is the expression of the transfer function (log sigmoid function), *e* takes the natural constant 2.718. The connection weight *ω*_*ji*_ mainly reflects the connection strength between the layers of BPNN, and when *ω*_*ji*_ exceeds 0, the function is activated. In addition, when the sample data volume is large, the convergence speed of BPNN is reduced, and the real-time performance of inhibition is poor. Therefore, the particle swarm optimization (PSO) algorithm with easy implementation and high convergence speed is studied to optimize BPNN [27].

If the particle swarm is composed of *m* particles, the different particles correspond to a feasible solution to the problem. The d-dimensional position vector of the *i* particle is expressed as *z*_*i*_=(*z*_*i*1_, *z*_*i*2_,…, *z*_*iD*_), the flight speed of the particle is expressed as *v*_*i*_=(*v*_*i*1_, *v*_*i*2_,…, *v*_*iD*_), the optimal position of the particle so far is expressed as *p*best_*i*_=(*p*_*i*1_, *z*_*i*2_,…, *p*_*id*_,…, *p*_*iD*_), and the optimal position of the whole particle swarm so far is expressed as *g*best_*i*_=(*g*_*i*1_, *g*_*i*2_,…, *g*_*id*_,…, *g*_*iD*_).

(5) $$\begin{array}{c} v_{i\;d}^{k+1}=WV_{i\;d}^{k}+c_{1}r_{1}\left(p_{id}-z_{id}^{k}\right)+c_{2}r_{2}\left(g_{d}-z_{id}^{k}\right), \end{array}$$

(6) $$\begin{array}{c} z_{id}^{k+1}=z_{id}^{k}+v_{id}^{k+1}. \end{array}$$

Equation (5) is the update expression of particle velocity, and equation (6) is the update expression of particle position where *k* and *W* represent iteration times and inertia weight in turn; *r*_1_ and *r*_2_ is a random number between [0, 1]; *c*_1_ refers to learning factor; and *c*_2_ is acceleration factor; usually, the empirical value is *c*_1_=*c*_2_=1. The current position of particles in the population can be expressed as the set of BP weights and thresholds. The neural network weight matrix and neural network threshold are scanned, and the particle position is initialized.

(7) $$\begin{array}{c} v_{i\;d}^{k+1}=\theta v_{id}^{k}+c_{1}r_{1}\left(p_{id}-z_{id}^{k}\right)+c_{2}r_{2}\left(g_{d}-z_{id}^{k}\right). \end{array}$$

According to equations (6) and (7) to complete the iteration,

(8) $$\begin{array}{c} \theta =\theta_{\max}-\frac{\theta_{\max}-\theta_{\min}}{k_{\max}}\times k. \end{array}$$

Formula (8) is the weight *θ* calculation formula of particle velocity iteration, where *θ*_max_ is the initial weight, *θ*_min_ is the final weight, *k*_max_ is the maximum number of iterations, and *k* is the current number of iterations. In the process of research, the PSO algorithm is used to train the weights and thresholds of BP neural network and then find out the optimal position of particle swarm optimization.

(9) $$\begin{array}{c} \omega_{i,j}^{k+1}=\omega_{i,j}^{k}+v_{i\;d}^{k+1}. \end{array}$$

Formula (9) is the learning formula of network weight and network threshold, where *v*_*id*_^*k*+1^ is the corresponding speed of particles in the *k*+1 iteration and *ω*_*i*,*j*_^*k*^ is the corresponding weight of particles in the *k* iteration.

(10) $$\begin{array}{c} y_{j,i}^{d}=\frac{1}{\left(1+e^{-\sum_{i=1}^{N}\omega_{ij}}\right)}. \end{array}$$

Equation (10) is the expression of the maximum fitness principle, where *y*_*j*,*i*_^*d*^ represents the ideal output value of the sample corresponding to the output node of the network, *ω*_*ji*_ represents the weight corresponding to the output node, and *N* is the number of network layers.

(11) $$\begin{array}{c} E\left(X_{i}\right)=g{\text{best}}_{i}\times \frac{1}{N}\sum_{i=1}^{N}\sum_{j=1}^{t}{\left(y_{j,i}^{d}-y_{j,i}\right)}^{2}. \end{array}$$

Equation (11) is the minimum principle expression of mean square error, where *t* is the number of neurons output by the network and *y*_*j*,*i*_ represents the actual value of the sample at the output node.

### 2.2. Construction of Safety Risk Evaluation Index System of Tourism Management System

With the improvement of science and technology, tourism practitioners gradually use the management system to manage tourism-related information, and the privacy information of tourism customers is recorded in the network. In order to ensure that the information of tourism customers is not infringed, it is very important to evaluate the security risk of the tourism management system. Based on PSO-BP neural network, according to the basic content of the tourism security management system, the system security risk evaluation index is determined.

As shown in Figure 2, according to the basic content of the tourism security management system, seven security risk indicators such as user personal information security risk index, information security risk index of scenic spot resources, hotel resource information security risk index, restaurant resource information security risk index, information security risk indicators of entertainment and shopping resources, risk indicators of traffic resource information security in the process of tourism, and tourism route information security risk index are selected as the main indicators affecting the security risk of the tourism management system.

Suppose that the parameter of security risk influencing factors of the tourism management system is expressed as *x*_*i*_(*i*=1,2,…, *m*), *k* experts are selected to score the corresponding security risk index, and the corresponding partition of the *h* expert is recorded as [*u*_1_^*k*^, *u*_2_^*k*^], where *u*_*i*_ ∈ [0,1].

(12) $$\begin{array}{c} \bar{u}=\frac{\sum_{h=1}^{k}\left[{\left(u_{1}^{h}\right)}^{2}-{\left(u_{2}^{h}\right)}^{2}\right]}{\sum_{h=1}^{k}\left[u_{1}^{h},u_{2}^{h}\right]}. \end{array}$$

Equation (12) can be used to evaluate the objectivity of safety risk index $\bar{u}$, where *u*_1_^*k*^ and *u*_2_^*k*^, respectively, refer to the lowest score and the highest score given by the *h* expert and *k* is the total number of experts involved in the evaluation.

(13) $$\begin{array}{c} b_{i}=\sum_{j=1}^{n}\frac{b_{ji}}{n}. \end{array}$$

Formula (13) is mainly used to calculate the reliability of the evaluation index. The total confidence of the safety risk index *x*_*i*_ is expressed as *b*_*i*_, and *b*_*ji*_=1/(1+*g*), where *g* is the safety risk identification index. When the evaluation risk is *j*, the confidence of *x*_*i*_ is expressed as *b*_*ji*_. Quantitative treatment is applied to the safety risk related indicators of the tourism management system, and the specific quantitative method is shown in Figure 3.

(14) $$\begin{array}{c} \left\{\begin{array}{c} g_{i}=\frac{1}{3}\frac{\sum_{h=1}^{k}\left[{\left(u_{1}^{h}-\bar{u}\right)}^{3}-{\left(u_{1}^{h}-\bar{u}\right)}^{2}\right]}{\sum_{h=1}^{k}\left[u_{1}^{h},u_{2}^{h}\right]},\\ x_{i}=\bar{u}b_{i}. \end{array}\right) \end{array}$$

In formula (14), *x*_*i*_ is the safety risk index and *k* is the total number of experts participating in the evaluation.

Through the expert evaluation method, different experts evaluate the security risk of the tourism management system according to their own actual cognition, including the overall evaluation. Combined with the experts' own experience, the grading of the comment set is determined.

As shown in Figure 4, the security risk equivalence of tourism management systems can be divided into five levels: Level 1–5. The corresponding risk levels are low risk, low risk, medium risk, high risk, and high risk. The scores for the different risk levels are [0.0, 0.2], [0.2, 0.4], [0.4, 0.6], [0.6, 0.8.], and [0.8, 1.0]. Training the sample data should be performed according to different risk levels.

As shown in Figure 5, the PSO-BP neural network is used to train the sample data of the security related risks of the tourism management system. The risk factors affecting the security of the tourism management system are taken as the input layer, and the security risk level of the tourism management system is taken as the output layer.

## 3. Application Effect Analysis of Security Risk Assessment of Tourism Management System Based on PSO-BP Neural Network

### 3.1. Application Effect Analysis of PSO-BP Neural Network Model

In order to verify the practical operation effect of the PSO-BP neural network and the actual operational effect of the PSO-BP neural network model designed in this study, 10,000 data related to the safety risk evaluation index of the tourism management system were selected as samples and 3,000 were randomly tested. And the other 7,000 are used as training samples.

Although limited by the length of the article, Figure 6 shows only the test results for some test samples. It turns out that the actual risk value of sample 1 is 0.3049, the risk value detected by the proposed PSO-BP neural network model is 0.4550, the actual risk value of sample 2 is 0.7731, and the risk value of the proposed model is 0.9233. The actual risk value for sample 5 is 0.2492, and the risk value detected in the proposed model is 0.2884. In summary, the risk values detected by the PSO-BP neural network model proposed in this paper are slightly higher than the actual risk values in the sample, but the difference between the two is not very large. In the experiment, the training sample and the test sample compare the error curve fitting graphs of the BP neural network algorithm and the PSO-BP neural network algorithm.

In Figure 7, the horizontal axis represents the number of sample iterations and the vertical axis represents the result of the curve error. It can be seen that when the number of iterations of the training sample reaches 600, the error result of the PSO-BP neural network algorithm tends to be 10–5, and the error result of the BP neural network algorithm is higher than 10–4. When the number of iterations of the test sample reaches 300, the error result of the PSO-BP neural network algorithm is close to 10–5, and the error result of the BP neural network algorithm is higher than 10–2. From the two error curves of the training sample and the test sample, we can see that under the same number of iterations, the error result of the BP neural network algorithm is always higher than the error result of the PSO-BP neural network algorithm.

From Figure 8, it can be seen that the average accuracy rate of the risk evaluation of the PSO-BP neural network algorithm proposed in this paper is 96.53% compared with the conventional BP neural network algorithm, which is significantly higher than that of the BP neural network. In terms of training time, the average training time of the PSO-BP neural network algorithm is 216 seconds, which is much shorter than the BP neural network algorithm (>10000 seconds). In terms of the number of iterations, the average PSO-BP neural network algorithm has 275 iterations, which is much less than the BP neural network. The average number of iterations (>18000) of the network algorithm is a relative error compared with the BP neural network algorithm. The PSO-BP neural network algorithm has a relative error of only 0.32%, and the BP neural network algorithm has a relative error of 0.45%. The above results show that the PSO algorithm can significantly reduce the convergence time and improve the convergence speed of conventional BP neural network algorithms. The final PSO-BP neural network algorithm has more powerful advantages than the traditional BP neural network algorithm.

### 3.2. Performance Analysis of Safety Risk Assessment Scheme

To compare the effectiveness of the proposed security risk assessment method for tourism management systems based on the PSO-BP neural network, the traditional security assessment technology for tourism management systems is compared with the proposed technology. The survey target is the security risk data set *X* of the tourism management system, and there are 200 samples in the survey target. In the experiment, 100 samples are randomly selected as test samples and the remaining 100 samples are used as training samples.

As shown in Figure 9, with the increase in the number of training samples, the training error of the proposed risk assessment method presents a decreasing trend. When the number of training reaches 5, the corresponding output error of the proposed risk assessment scheme has been reduced to 10^−3^, reaching the preset range of convergence error. After the training of sample data, the weight value of evaluation index is determined.

According to Figure 10, the corresponding weight values of user personal information security, tourism route information security, traffic resource information security, entertainment and shopping information security, restaurant resource information security, scenic spot resource information security, and hotel resource information security are 0.4, 0.15, 0.15, 0.15, 0.05, 0.05, and 0.05. According to the weight values corresponding to the above different safety risk indicators, the risk levels of different indicators are determined.

From Figure 11, the system safety risk value curve obtained by the risk evaluation method of the proposed PSO-BP neural network-based tourism management system is almost in agreement with the actual risk value curve and is in line with the conventional system. We can see that there is a big error in safety risk curve and actual risk curve. In other words, the risk assessment method of the tourism management system based on the PSO-BP neural network proposed in this study is more accurate and effective in the security risk assessment of the tourism management system. The security risk assessment of the tourism management system is mainly the system information risk assessment. Therefore, we selected a security risk evaluation model based on fuzzy sets and entropy weighting theory and an information system security risk evaluation model based on gray correlation analysis and radial basis function neural networks as comparison targets, and the effects of applying the three methods are as follows. Information system security risk assessment methods include the methods proposed in Dataset *X*. For each program, 20 experiments were performed and average values were taken.

As shown in Figure 12, the average evaluation accuracy of the security risk evaluation model based on the fuzzy set and entropy weighting theory is 96.90%. The average evaluation accuracy of the information system security risk evaluation model based on neural network is 96.90% and the average evaluation accuracy rate of the evaluation scheme based on the PSO-BP neural network is 99.72%. The average time for risk assessment based on fuzzy sets and entropy weighting theory is 2.593 seconds, and the average time for security risk assessment of information systems based on gray relation analysis and radial basis function neural networks is 3.081 seconds, based on only 2.512 seconds. The above results are compared with the security risk assessment scheme based on fuzzy set and entropy weighting theory and the information system security risk assessment scheme based on gray relation analysis and radial basis function neural network, and the tourism security risk assessment proposed in this paper. The results show that the neural network management system based on PSO-BP has the advantages of high evaluation accuracy, short calculation time, and excellent safety risk evaluation performance.

## 4. Conclusion

Traditional tourism management system security risk assessment schemes have the disadvantage of causing large assessment errors when performing system security risk assessments. Therefore, this paper uses particle swarm optimization (PSO) to improve the slow convergence rate of traditional BP neural networks and is prone to local optimal solutions and the security risks of tourism management systems based on PSO-BP neural networks. We propose evaluation technology. The convergence time of the BP neural network algorithm, which can be shortened, improves the accuracy of risk value assessment. The results show that under the same number of iterations, the error results of the proposed PSO-BP neural network are always smaller than the error results of the traditional BP neural network. If the test sample is repeated 300 times, the error result is that the error in the PSO-BP network is close to 10–5. The error results for the BP network are still higher than 10–2, the average accuracy for the PSO-BP network is high (96.53%), and the average training time is short (216 seconds); the number of iterations required (275) is relatively small, the error is small (0.32%), 87.21%, >10000 seconds, >18000 times, 0.45% better than traditional BP networks, respectively. The user's personal information security risk value is highest at 0.4, followed by tourist route information security and traffic resource information security. The risk value curve of the proposed risk assessment scheme is similar to the actual risk value curve. In summary, the proposed security risk assessment scheme for tourism management systems based on PSO-BP neural networks can effectively assess the security risks of tourism management systems. While this study has some value in how to improve the effectiveness of security risk assessments in tourism management systems, this scheme can only assess the value of risks and will continue to resist network intrusions. 

## Figures and Tables

**Figure 1:** Schematic diagram of BP neural network.

**Figure 2:** Security risk index system of the tourism management system.

**Figure 3:** Quantification of security risk identification index of the tourism management system.

**Figure 4:** Security risk assessment level of the tourism management system.

**Figure 5:** The steps of safety risk assessment of the tourism management system based on PSO-BP neural network.

**Figure 6:** Value at risk prediction results of test samples (part).

**Figure 7:** Comparison of error curves of two algorithms; (a) comparison of error curves of training samples; (b) comparison of error curves of test samples.

**Figure 8:** Comparison of simulation results of test samples. (a) Training time and iteration times of the two algorithms. (b) The average accuracy and relative error of the two algorithms are compared.

**Figure 9:** Training sample error.

**Figure 10:** The weight of the safety risk evaluation index of the tourism management system.

**Figure 11:** Comparison results of two methods in evaluating errors.

**Figure 12:** Comparison results of two methods in evaluating errors. Note: I refers to a security risk assessment model based on fuzzy sets and entropy weighting theory. II is an information system security risk assessment model based on gray correlation analysis and radial basis function neural networks. III represents the evaluation scheme based on PSO-BP neural network.

## Data Availability

The data used to support the findings of this study are available from the corresponding author upon request.
